This article has been retracted.

# Regional Differences and Convergence of Urban-Rural Integration Development from the Perspective of Factor Flow

**DOI:** 10.1155/2022/2695366

**Published:** 2022-08-22

**Authors:** Li Qian, Ke Zhang, Jun-Xiu Song, Wei-Yi Tang

**Affiliations:** ^1^School of Economics, Anhui University of Finance & Economics, Bengbu, Anhui 233030, China; ^2^School of Finance and Public Administration, Anhui University of Finance & Economics, Bengbu, Anhui 233030, China

## Abstract

Based on the panel data of thirty-one provinces in China from 2003 to 2020, we constructed an evaluation index system of urban-rural integration development level from the perspective of factor flow. The combined weighting model of GI and CRITIC were used to evaluate the regional urban-rural integration development. The coefficient of variation and panel fixed effect model was used to explore convergence, absolute convergence, and conditional convergence. The impact of capital, labor, and technology factor flow on the convergence of urban-rural integration development level was further investigated. In addition, the difference analysis in time scale and impulse response function analysis was performed to explore the regular pattern of factor flow on the convergence of urban-rural integration development. The main conclusions were as follows: first, the growth of urban-rural integration development had an absolute convergence trend and tended to conditional convergence faster. Second, the capital flow positively affected the convergence of urban-rural integration development, while labor and technology flow had a slowing effect on the convergence of urban-rural integration development at this stage. Third, the impact of factor flow on the convergence of urban-rural integration development was dissimilar during different phases. The convergence rate of urban-rural integration development after 2012 was drastically slower than before.

## 1. Introduction

The urban-rural disparity is a critical headspring of social structure differences. For a long time, “Urban bias” has existed and been popular due to people's wrong concepts and restrictions of development. In recent years, problems have become more and more apparent, like the gap between rural and urban economic development is increasingly widening, and the rural economy has been aggravating in some areas. The proportion of urban population and output rises due to the “Siphoning effects.” Agriculture has languished and lost development vigor, and rural areas face the issue of growing depopulation [1]. The economic policy of urban-rural division may appear lose-lose situation. In order to change the current situation of unbalanced urban and rural development, we should fundamentally solve problems concerning the relationship between urban and rural areas. We should accord the construction of the rural regions the same important position as the construction of the urban areas to motivate rural development. Based on this, considering China's reality and the current situation of rural development, this paper puts forward a rural revitalization strategy to make the government and market resource allocation at total capacity, promote the flow and equal exchange of urban and rural resources, and realize the purpose of urban-rural integration.

One of the important performances is the unbalanced development between urban and rural areas and inadequate development in rural areas. Promoting the integrated urban-rural development is the key to alleviating the unbalanced and inadequate development between urban and rural areas and the objective requirement of ensuring common prosperity between urban and rural residents. Urban and rural integration breaks the contrary state of the urban-rural dual structure and gradually realizes the rational flow and optimal combination of factors in urban and rural areas. Urban-rural coordinating development had been proposed as a strategy as far back as 2002. “Promote the integration of urban and rural development” was proposed in 2012. Furthermore, on this basis, integrated urban and rural development was proposed in 2017, emphasizing the interaction of urban and rural factors. The evolution of the policies might fully embody the development of cognition on urban-rural relations [2]. Urban-rural integration is an organic unity of factor allocation and public resources between urban and rural areas. The goal is to create a new shared urban-rural life community. However, urban-rural integration development in various regions is alienated due to different industrial policies, resource endowment, and other factors. Accordingly, urban and rural development would form a positive interaction in areas with a high level of urban-rural integration. There are few urban-rural links in districts with lower urban-rural integration levels, which causes widened gaps of development among regions. If significant regional gaps exist in the regional urban-rural integration development, the efficiency of integrated urban and rural development might be affected, which is not conducive for the efficient allocation of resources and the sustainable development of integrated urban-rural integration, contributes to the differences in income distribution and social welfare between regions, impacts the stabilization of the social order, which further impedes competition, efficiency, and shared prosperity. Therefore, a study on the growing convergence of urban-rural integration development and the integral grasp of regional urban-rural integration might play critical roles in weakening class distinction, narrowing the economic development gap among regions, and formulating related regional development policies.

Factor mobility between urban and rural areas might change the fundamental structure of urban and rural elements, influence the evolution of urban-rural relations, and then affect urban-rural integration development. At the micro-level, factor flow might put idle resources to work, promote balanced marginal returns growth in urban and rural elements, and realize complementary functional advantages and maximization of integral benefit [3]. At the macro level, labor, capital, and technology are crucial elements for the production-possibility frontier, improving efficiency and resource allocation. The urban-rural segmentation has long existed in China. In this regard, it seems to urge the rapid development of our country's economy. However, on the other hand, it restricts the development of agriculture in rural areas. In general, the resource elements have a unidirectional flow from rural to city, making urban-rural dual-element more and more emphasized. There is a severe imbalance in the allocation of urban and rural resources, and massive room for Pareto improvement remains in feature configuration. If the resource could be moved around more freely, the income between urban and rural areas will finally converge, and then the level of urban and rural development might gradually reach equilibrium. To crack the binary structure and overcome institutional barriers in the free flow of urban and rural elements, we should establish a new pattern of two-way flow, regulate the imbalance in the allocation of urban and rural resources, and provide further dividends for China's economic development.

## 2. Literature Review

Along with the development of urban-rural relations, the concept of urban-rural integration is continually developed [4]. Furthermore, its diversity and complexity determine that urban-rural integration is a multi-dimensional convergence [5]. Based on the richness of urban-rural integration, the criteria for evaluating the development level of urban-rural integration show a vast difference in evaluation index systems. Some scholars come up with the idea of constructing an evaluation index system for integrated urban-rural development based on the premise of three layers: development, motivator, and resultant factors [6]. Some academics establish a multi-dimensional index measurement system of “Population-Space-Economy-Society-Environment” based on the increasingly spatial connection between urban and rural areas [7]. Some academics put forward an analytical framework of urban-rural correlation symbiotic development based on urban-rural interaction and integration [8]. In addition, the regional heterogeneity of integrated urban-rural development was taken into consideration. They construct the dimension index system of urban and rural development and coordination [9]. The gravity model, geographic detector model, and bivariate VAR model are used to explore the impact of factors such as spatial aggregation [10] and financial services [11] on the development of urban-rural integration. On this basis, some researchers deeply study the development path of urban-rural integration, put forward that the social division of labor is the root of urban-rural confrontation [12].

In recent years, the study on the flow of urban and rural factors has been roughly divided into three aspects [13]. Some studies explore the relationship between factor flow and urban-rural integration development [14]. They suggest that the connotation of urban-rural integration includes the free flow and rational allocation of urban-rural factors [15], which have spawned the optimal allocation of value-added income. However, in the process of rapid urbanization and industrialization, the long-term “nonagricultural bias” leads to the “loss” of rural traditional production factors [16], which increases the dependence of rural areas on cities in employment, medical treatment, education, and other aspects [17]. Furthermore, some researchers began to focus on the internal logic of factor mobility and urban-rural integration. They find that the loosening effect of household registry reform on labor mobility and the circulating effect of city industry for high-quality talents might change the objective function of individuals and achieve the convergence of urban and rural social economy [18]. Capital flows from the initial profit to the urban industrial sector and then overflows from the city to the countryside under the aggregation-dispersion mechanism due to the impact of congestion cost on the urban economies [19]. The rapid development and improvement of the intercity transportation networks and information networks promote the formation of urban agglomeration, strengthens the industrial agglomeration effect of urban agglomeration, and accelerates urban technological innovation. Moreover, the rise of intercity land price and inflation promote the extension of the industry to rural areas and accelerate the sharing and renewal of technology between urban and rural areas [20]. In addition, other studies explore the dilemmas, mechanisms, and countermeasures of urban and rural factor mobility under the background of enhanced factor mobility. There are still some problems in the flow of urban and rural factors, such as unsmooth flow and unreasonable flow direction, and no trend of narrowing the income gap between urban and rural areas.

It is normal to have a certain degree of development gap in social and economic development [21, 22]. However, the persistence or widening trend of the gap is not conducive for the development of the economy and the effective allocation of resources [23]. Therefore, it is necessary to study the problem of convergence. Recently, most studies on convergence concentrate on the gap and junction of the regional economy, and other research has shown the convergence of new urbanization growth [24]. However, the study on the regional gap and growing convergence of urban-rural integration development remains insufficient. The only relevant studies focus primarily on qualitative research; simultaneously, the empirical analysis and the impact of factor flow on the growing convergence of urban-rural integration development remain largely elusive. We should promote urban-rural integration and prevent the expansion of the development gap between regions caused by the difference in urban-rural integration development. Therefore, it is essential to carry out a study on the regional differences and growing convergence of urban-rural integration development, to improve the quality of urban-rural integration development. This is conducive for the precise implementation of urban-rural integration in the future.

In short, other studies on the overall development of urban and rural areas and their index systems cover three dimensions: society, economy and ecology, mainly adopting the ratio of urban and rural indicators, and then making a descriptive analysis of the results. The research on the combination of urban-rural integration and factor flow focuses on the internal logic and relationship, lacking specific empirical research. The possible marginal contributions of this paper are as follows: Firstly, given that urban and rural areas are two different social forms, the state indicators and dynamic indicators showing the integrated of urban-rural development are added on the basis of the mainstream of urban-rural comparative indicators in the past; the spatial integration dimension is added to the indicator system for the closer spatial connection between urban and rural areas. Secondly, from the perspective of factor flow, this paper analyzes the regional gap and convergence of the integrated urban-rural development. It also further explores the differences of labor, technology, and capital factor flow on the integrated urban-rural development convergence, which not only provides reference for further promoting integrated urban-rural project but also provides theoretical support for guiding the free and orderly flow of factors. Thirdly, by means of using provincial data, this paper examines the distribution and convergence of the overall integrated urban-rural development at a macro level, and explores the influence of the flow of factors between urban and rural areas in different provinces on the overall integrated urban-rural development and regional economy.

## 3. Theoretical Analysis

### 3.1. Convergence of Factor Flow to Urban-Rural Integration Development

From the perspective of spatial evolution, the difference of factor resource endowment between urban and rural areas is the initial reason for the low level of urban-rural integration development. With the advancement of industrialization, the centripetal force formed by the city's market effect and price index effect makes the factors gather in the urban area, which gradually improved the production conditions and quality of life in urban area. The flow of factors promotes rapid urban economic growth. At the same time, this process also accelerates the process of element agglomeration. Once the accumulation of factors in urban reached a specific size, the cost of living and production in cities is gradually rising, which might create centrifugal forces and crowding effect, and progressively transfer factors to rural areas, promote rural economic development, narrow the development gap between urban and rural areas, and improve the development level of urban-rural integration. By promoting the two-way flow of urban and rural factors in various regions, urban-rural integration development gradually balances. Finally, the convergence of urban-rural integration is realized. Our growth function of urban-rural integration development level is as follows:

(1) $$\begin{array}{c} \ln\;y_{t+1}^{i}-\ln\;y_{t}^{i}=f\left\{y_{t}^{i},g_{t}^{i}\left(L_{t}^{i},K_{t}^{i},A_{t}^{i}\right),x_{t}^{i}\right\}. \end{array}$$

As shown in the above formula, the growth of urban-rural integration development level (ln  *y*_*t*+1_^*i*^ − ln  *y*_*t*_^*i*^) is affected by the urban-rural integration development level (*y*_*t*_^*i*^) of the region and the gap between areas (*g*_*t*_^*i*^(*L*_*t*_^*i*^, *K*_*t*_^*i*^, *A*_*t*_^*i*^)) and other factors (*x*_*t*_^*i*^). The gap between areas is affected by the stock and flow of labor, capital, and technology. Based on this, Hypothesis 1 is proposed in this study.

  H1: factor flow might play a critical role in converging urban-rural integration development.

### 3.2. Convergence of Different Factor Flows on Urban-Rural Integration Development

Urban and rural elements are divided into the labor force, capital, technology, and land according to production factors when they flow. Labor, capital, and technical factors flow more actively between urban and rural areas. Specifically, the reform of the registered residence system promotes the flow of rural surplus labor to cities. To gain circulation effect among high-quality labors, city industries have changed individual objective function. By doing this, they expect to achieve the convergence of urban-rural economy and promote the balanced integrated urban-rural development. Due to its profit-seeking nature, capital flows to the industrial sector in the city. After forming a specific scale, it is affected by the crowding effect. Under the aggregation-dispersion mechanism, capital elements overflow from the city to the countryside. The rural economy gradually recovers, promoting the integration of urban and rural industries and urban and rural integration. With the rapid development of intercity transportation and information network, the economic scale effect of urban agglomeration is strengthened. Urban technological innovation is accelerated while promoting the formation of urban agglomeration. Moreover, the rise of intercity land price and inflation might encourage the extension of the industry to rural areas and the sharing and upgrading of technology between urban and rural areas, promoting the balanced growth and development of urban-rural integration. This study further explores the internal relationship between the flow of labor, capital, and technology factors and the growth and convergence of urban-rural integration development. The transfer equations of labor, capital, and technology are as follows.

#### 3.2.1. Labor Transfer Equation

A model with two regions is considered. Suppose there are skilled and unskilled labor groups in both regions, denoted as *H*, *L*, and the corresponding natural growth rate is *h*, *n*. During the actual flow of factors, its scale depends on the marginal income gap of related factors between regions. Whether labor force across regions can be transferred or not only depends on wage differences of homogeneous labor force in different regions. The dynamic accumulation equations for the labor factors of the region *i* are as follows:

(2) $$\begin{array}{c} H_{t+1}^{i}=\frac{\left(1+h\right)H_{t}^{i}+WH_{t}^{i}-WH_{t}^{i}}{WH_{t}^{s}\left(1-H_{t}^{i}+\left(L_{t}^{i}/N_{t}^{i}\right)\right)H_{t}^{n}},\;i\neq j, \end{array}$$

(3) $$\begin{array}{c} L_{t+1}^{i}=\frac{\left(1+n\right)L_{t}^{i}+WL_{t}^{i}-WL_{t}^{j}}{WL_{t}^{s}\left(1-H_{t}^{i}+\left(L_{t}^{i}/N_{t}^{i}\right)\right)L_{t}^{n}},\;i\neq j. \end{array}$$

The above formula (1 + *h*)*H*_*t*_^*i*^ indicates the natural growth (*WH*_*t*_^*i*^ − *WH*_*t*_^*j*^/*WH*_*t*_^*s*^) and suggests the transfer ratio caused by the reward gap of *H* factors between regions. The scale of labor mobility increases with the increase of the pay gap. However, there is an upper limit on labor transfer. The congestion function is defined as *m* = *H*_*t*_ + (*L*_*t*_/*N*_*t*_)*N*_*t*+1_ = (1 + *φ*)*N*_*t*_, indicating that the regional population capacity limits the proportion of labor mobility. Similarly, the meaning of the labor mobility equation is similar to that of *H*. When the pay gap between regions of *H* factor is higher than that in *L*, its proportion of labor transfer is also higher. With the increase *H*, the scale of subsequent labor flow is limited in places of influx and finally the number of *H* and *L* reaches a balance in the process.

Due to the development gap between regions, labor wages are created, promoting the transfer of labor force, and the regional crowding effect crowding out unnecessary labor force. Promoting the free and orderly flow of the labor force might affect the regional development gap. Based on this, hypothesis 2a is proposed in this study.

  H2a: labor mobility plays a crucial role in converging urban-rural integration development.

#### 3.2.2. Capital Transfer Equation

The capital transfer is affected by the differences in regional interest rates. It is worth noting that fixed and new capital transfer speed is different. It is assumed that the transfer proportion of new capital *g*_*k*_*K*_*t*_ is entirely determined by the interest rate difference between regions (the ratio is (*R*_*t*_^*i*^ − *R*_*t*_^*j*^)/*R*_*t*_^*s*^). The former fixed capital transfer is multiplied by the realization coefficient *t* based on this proportion. Therefore, the simplified form of capital transfer equation is as follows:

(4) $$\begin{array}{c} K_{t+1}^{i}=\left(1+g_{k}\right)K_{t}^{i}+\left(t+g_{k}\right)\left(\frac{R_{t}^{i}-R_{t}^{j}}{R_{t}^{s}K_{t}^{n}}\right),\;i\neq j. \end{array}$$

As shown in the above formula, when the interest rate in region *i* is lower than in region *j*, the item (*R*_*t*_^*i*^ − *R*_*t*_^*j*^) becomes negative. Currently, the elements in the *j* area show a trend of backflow. Affected by the difference of interest rates between regions, the capital flow might promote the capital flow, which affects both the regional economic development and the urban and rural integration and development. Based on this, hypothesis 2b is proposed:

  H2b: capital flow has a critical impact on the convergence of urban-rural integration development.

#### 3.2.3. Technology Transfer Equation

Technology transfer is affected by the proportion of science and technology funds in financial expenditure (the rate of technology investment). Like the above capital transfer equation, the simplified form of the technology transfer equation is as follows:

(5) $$\begin{array}{c} A_{t+1}^{i}=\left(1+g_{a}\right)A_{t}^{i}+\left(t+g_{a}\right)\left(\frac{T_{t}^{i}-T_{t}^{j}}{T_{t}^{s}A_{t}^{n}}\right),\;i\neq j. \end{array}$$

The setting of the above formula does not limit the inflow and outflow places. When the interest rate of region *i* is lower than the regional technology input rate of region *j*, (*T*_*t*_^*i*^ − *T*_*t*_^*j*^), it becomes negative. The elements of the *j* area show a return trend. Affected by the difference in technology input rate, technology flows between regions, affecting regional economic development and urban-rural integration development. Based on this, hypothesis 2c is proposed:

  H2c: technology flow has a crucial impact on the convergence of urban-rural integration development.

Based on the abovementioned, promoting the integrated urban-rural development is actually promoting the two-way flow of elements between urban and rural areas. For a long time, a large number of productive factors in rural areas have continuously flowed into cities unidirectionally, resulting in serious “blood loss” in rural areas. In the new relationship between urban and rural areas, rural elements flow to cities, and urban elements also flow to rural areas, which will form a virtuous circle of two-way flow of urban and rural elements. It is essential to guide the factors to flow freely and orderly between urban and rural areas, and activate the endogenous power of rural development through “optimizing the combination effect of factors,” “spillover effect of knowledge dissemination technology,” and “expanding market scale effect by division of labor,” so as to promote the integrated development of urban and rural areas.

## 4. Research Design

### 4.1. Description for Variables

#### 4.1.1. Explained Variable

The growth level of urban-rural integration development. Based on Chang et al. [25], the difference between the current and lagging levels of urban-rural integration development is used to measure the growth level of urban-rural integration development. Whether it is “urban-rural equivalence” from the perspective of foreign factor flow or multi-dimensional integration and interaction between urban and rural areas in the process of domestic regional development, it will eventually turn from “heterogeneous dual structure” to “homogeneous integration,” which is the key to the integrated development between urban and rural areas. On the construction of the index system of the integrated urban-rural development, based on the existing related research and the rich connotation of the urban-rural development, the construction not only includes the comparative index reflecting the urban-rural difference but also includes the development degree index showing the “urban-rural development community” from the five dimensions, such as “society,” “economy,” “ecology,” “culture,” and “space,” which is shown in Table 1.

#### 4.1.2. Core Explanatory Variables

Development level of urban-rural integration, labor flow, capital flow, and technology flow. The development level of urban-rural integration is measured by establishing an index system and calculating the urban-rural integration development index. We construct an evaluation index system for urban-rural integration development, following the scientific and creative principles. Labor flow equals the ratio of the number of employees in this province and the average number of employees in other regions in the current year. Capital flow equals the balance of the number of capital formation rates to the average value of capital formation rate in the current year in other provinces. Technology flow equals the ratio of this province's science and technology expenditure (R&D expenditure) to the average science and technology expenditure of other regions.

#### 4.1.3. Control Variables

Per capita GDP (logarithm), fiscal decentralization, and rural financial services in this region. The higher the regional GDP, the better the regional economic development, which could drive regional urban-rural growth and impact urban-rural integration development. The higher the level of fiscal decentralization, the more autonomy the local government has, which could reasonably arrange urban and rural resources, promote resource allocation, and promote regional urban-rural integration and development. Rural financial services mean financial support for rural areas. The more thoughtful rural financial services are, the more funds might be provided for rural development, which could accelerate the speed of urban-rural integration and development. The above control variables are measured by the proportion of local government income in total income and per capita agriculture-related loans (logarithm).

### 4.2. Specification of the Model

#### 4.2.1. *β* Convergence Model

The econometric model selected in this study refers to the research on the setting of the convergence model by Bakbak and Kansu [26] and Cholamjiak and Baiya [27]. The following model is used to evaluate whether the growth of urban-rural integration development level is convergent.

(6) $$\begin{array}{c} \left(\frac{1}{T}\right)\ln\left(\frac{y_{i,t}}{y_{i,t-T}}\right)=\alpha -\ln\left(\frac{\left(y_{i,t-T}\right)\times \left(1-e^{-\beta T}\right)}{T+Z}\right). \end{array}$$

Among them, *y*_*i*,*t*_ is the development level of urban-rural integration in the region *i* during the period*t*, *y*_*i*,*t*−*T*_ is the development level of urban-rural integration in the region *i* at the beginning of the interval*T*. Due to the short observation period, this study investigates the growth rate of urban-rural integration development in one (1/*T*)ln(*y*_*i*,*t*_/*y*_*i*,*t*−*T*_) year. The average annual growth rate of the development level of urban-rural integration in the region *β* is the convergence rate of the development level of urban-rural integration in the region. Variable *Z* includes fiscal decentralization, rural financial services, industrial structure, and other factors that might affect the growing convergence of urban-rural integration development. At the same time, to avoid simultaneous errors of variables, we deal with the first-order lag of critical investigation variables and control variables.

According to formula (6), the following econometric model is established to evaluate the impact of factor flow in different provinces on the convergence of urban-rural integrated development from the proposal of “coordinating urban-rural economic and social development” in 2002. The specific form is as follows:

(7) $$\begin{array}{c} \ln\;y_{i,t}-\ln\;y_{i,t-1}=m_{0}+m_{1}\ln\;y_{i,t-1}+m_{2}\ln\;K_{i,t-1}+m_{3}\ln\;y_{i,t-1}\times \;\ln\;K_{i,t-1}+\phi X_{i,t-1}+\mu_{i}+v_{t}+\xi_{i,t}. \end{array}$$

ln  *y*_*i*,*t*_ − ln  *y*_*i*,*t*−1_ refers to the growth of regional urban-rural integration development level in the year; *y*_*i*,*t*−1_ is the development level of urban-rural integration that lags behind the first stage; *K*_*i*,*t*−1_ is the factor flow that lags behind the first period in the region, including labor flow lm, capital flows *cf*, technology flow *tf*; *X*_*i*,*t*−1_ is a series of control variables that affect the growth of regional urban-rural integration development; *u*_*i*_ refers to the individual effect; *v*_*t*_ indicates the time effect; *ξ*_*i*,*t*_ is a perturbation term.

#### 4.2.2. Convergence Model

The *σ* convergence model belongs to the concept of convergence in neoclassical economic growth theory. If there is *σ* convergence in the level of urban-rural integration, then the urban-rural integration converges in absolute value and finally realizes the balanced development of urban-rural integration. The coefficient of variation was used to measure the convergence of urban-rural integration, as shown in the following formula:

(8) $$\begin{array}{c} \sigma =\frac{\text{SD}}{MN}. \end{array}$$

Values were expressed as mean ± SD.

### 4.3. Data Sources and Descriptive Statistics

The data used in this study are from the relevant years of «China Financial Statistics Yearbook», «China urban and rural construction statistics yearbook», provincial statistical yearbooks, EPS database (https://olap.epsnet.com.cn, accessed on December 16, 2021)). Some missing data are supplemented by interpolation. Due to the lack of data from Hong Kong, Macao, and Taiwan, 31 provinces and cities are selected as the research objects. The following table is the basic descriptive statistics for the samples. To avoid the objective deviation caused by experts' subjective judgment and incomplete data statistics and make up for the lack of single weighting, we adopt the combination of the G1 method and critical subjective and objective weighting method. Taljaard and Mare [28] calculated the total weight by equally weighted averaging. The results are shown in Table 2.

As shown in Table 2, in social integration, the significant standard deviation of urban and rural endowment insurance coverage indicates the discrete degree of data, of which the maximum value is 97.460%, and the minimum value is only 8.900%. In economic integration, the maximum difference between urban and rural fixed investment is 4085.607, the minimum value is 5.156, and the average value is 117.418, suggesting that the deviation of test data is significant. In ecological integration, the standard deviation of solid waste production is as high as 9558.504, suggesting significant differences in the solid waste production among provinces and cities. In the process of cultural integration, the highest number of township cultural stations in various provinces and cities is 4641, and the least is 86. The degree of cultural transmission varies among regions; in spatial integration, the standard deviation of urban spatial expansion is also significant. The standard deviation of technology flow is more considerable than labor flow and capital flow [29]. These results implied that the difference in technology flow among provinces and cities is more significant than other factors.

## 5. Empirical Analysis

### 5.1. *β* Convergence Model Validation

In the benchmark regression, the coefficient of variation and benchmark regression were used to verify the absolute convergence; then, the influence of factor flow on the growing convergence of regional urban-rural integration development was evaluated by introducing the interaction term between factor flow and the initial urban-rural integration development; finally, a series of variables that might affect the convergence of urban-rural integration development is employed as control variables to further assess the robustness of the above results, including fiscal decentralization (L. fd), rural financial services (L. lnrfs), and per capita GDP (L. lnpgdp). Before the empirical analysis, the unit root inspection was carried out on the panel data, and the results demonstrated that the variables were stable. There are three models for panel data model estimation: mixed regression model, fixed-effect model, and random effect model [30, 31]. The mixed estimation is unsuitable for this study because there are apparent differences in urban-rural integration development and factors among individuals from different provinces and cities. Finally, the Hausman test was performed, and the results indicated that the *p* value = 0, rejecting the original hypothesis of random effect. The fixed-effect model estimation of panel data was selected based on this data.

#### 5.1.1. Absolute *βC* Convergence Model

The fixed effect was estimated for the panel data to validate whether there was absolute convergence of the development level of urban-rural integration. The benchmark regression results are exhibited in Table 3.

As shown in Table 3, the regression coefficient of L. lny in the model (1) was negative, indicating that there was absolutely a *β* Convergence trend in the growth of urban-rural integration development in China with provinces and cities as samples by using the fixed effect estimation of panel model *β*. After controlling the time effect in model (2), the coefficient of L. lny was still negative, indicating that this result was relatively robust. After adding variables such as fiscal decentralization (FD), rural financial services (Lnrfs), and per capita GDP (lnpgdp), the regression coefficient of L. lny was still negative regardless of whether the time effect was controlled. The convergence rate in model (3) was 0.087 percentage points higher than that in model (1), and that in model (4) was 0.053 percentage points higher than that of model (2). These data indicated a trend of absolute convergence in the growth of regional urban-rural integration development. Moreover, this growth might tend to conditional convergence at a faster speed.

#### 5.1.2. *βC* Conditional Convergence Model

We next investigate the convergence of factor flow on the growth of urban-rural integration development, the interaction terms of capital flow and urban-rural integration development, labor flow and urban-rural integration development, technology flow, and urban-rural integration development were introduced into the model, respectively. The benchmark regression results are shown in Table 4.

As shown in Table 4, models (9) and (10) considered labor mobility. After introducing the interactive term between labor mobility and urban-rural integration development, the coefficient of urban-rural integration development in the base period, the coefficient of labor mobility, and the coefficient of the interactive term were negative, indicating that labor mobility could decrease the development of urban-rural integration. Moreover, labor mobility could affect the convergence of the growth of urban-rural integration development through the interaction effect with urban-rural integration. Specifically, compared with model (1), the coefficient of L. lny in model (9) decreased from 0.036% to 0.021%, indicating that labor mobility had a slowing effect on the growing convergence of urban-rural integration development. For every 1% increase in capital flow, the convergence rate of regional urban-rural integration development decreased by 0.5% 015% ( = 0.036%–0.021%). After considering the time effect and introducing control variables in the model (12), compared with the model (4), the convergence rate of urban-rural integration development still decreased, indicating that the results are more robust and thus confirming hypothesis 2a.

As shown in Table 5, models (5) and (6) considered capital flow. After introducing the interactive term between capital flow and urban-rural integration development, the coefficient of urban-rural integration development in the base period was negative. The coefficient of capital flow and the coefficient of the interactive term were positive, indicating that capital flow might promote the growth of urban-rural integration development. Moreover, the capital flow might affect the growing convergence of urban-rural integration development through the interaction effect with urban-rural integration development [32]. Specifically, compared with model (1), the coefficient of l. lny in the model (5) increased from 0.036% to 0.093%. This result indicated that capital factor flows positively affected the growing convergence of the urban-rural integration development level. Specifically, for every 1% increase in capital flow, the convergence rate of regional urban-rural integration development increased by 057% (=0.093%–0.036%). However, after considering the time effect, the convergence rate of regional urban-rural integration development still rose, indicating that conditional convergence might ensure that the gap between backward and advanced areas of urban-rural integration does not get larger. After introducing a series of control variables such as fiscal decentralization (FD), rural financial services (Lnrfs), and per capita GDP (lnpgdp), the impact of capital flow on the convergence of urban-rural integration had not changed substantially, indicating that the results were relatively stable, and thus confirmed hypothesis 2b.

As shown in Table 6, models (13) and (14) considered technology flow. After introducing the interactive term of technology flow and urban-rural integration, the coefficient of urban-rural integration development in the base period, the coefficient of technology flow, and the coefficient of the interactive term were negative, indicating that technology flow also had a slowing effect on the development speed of urban-rural integration. At the same time, technology flow could affect the convergence of urban-rural integration development through interacting with urban-rural integration. Specifically, compared with model (1), the coefficient of L. lny in model (15) decreased from 0.036% to 0.026%, indicating that capital factor flow influenced the growing convergence of urban-rural integration. For every 1% increase in technology flow, the convergence rate of regional urban-rural integration development increased by 0.010% ( = 0.036%–0.026%). After considering the time effect and introducing a series of control variables in model (16), compared with the model (4), the convergence rate of urban-rural integration development still decreased by 0.007 percentage points. These stable results confirmed hypothesis 2c. In the end, these results might confirm hypothesis 1.

### 5.2. *σC* Convergence Model Verification

Before the *σ* convergence verification, we first understood the improvement process of regional urban-rural integration development. Here, we depicted the density diagram of urban-rural integration development before and after the year of the promulgation of the policies of “coordinating urban-rural economic and social development,” “promoting urban-rural integration,” and “urban-rural integration.”

As shown in Figure 1, in 2003, 2012, 2017, and 2020, the upgrading process of urban-rural integration development in various provinces and cities significantly altered, which is reflected explicitly in the rapid shift of the peak to the right year by year, indicating that the urban-rural integration development of various provinces and cities exhibited an overall upward trend, and the upgrading process were comparatively fast. In 2020, the wave crest of integrated development slightly reduced, whereas the left tail end slightly raised, indicating that the gap between regional urban and rural integrated development might be widened. The absolute convergence (*σ* convergence) of regional urban-rural integration development and factor flow was measured by the variation coefficient of urban-rural integration development and factor flow. As shown in Figure 2, the growth of urban-rural integration development in all provinces and cities from 2003 to 2020 had overall absolute convergence (*σ* convergence). The coefficient of variation of factor flow was greater than that of urban-rural integration. From big to small, the coefficient of variation of factor flow among provinces and cities was technology flow, labor flow, and capital flow [33].

## 6. Further Analysis

### 6.1. Period Difference Analysis

Affected by the implementation of the policy, the impact of factor flow on the growing convergence of the development of urban-rural integration in provinces and cities might be diverse during different phases. After the proposal of “coordinating urban-rural economic and social development” in 2002, the relationship between urban and rural areas had changed from Urban-Rural separation to urban-rural integration. “Promote urban-rural integration” was proposed in 2012. It is reasonable to believe that there might be pronounced period heterogeneity in the impact of factor flow on the growth of urban-rural integration development in different provinces and cities. It is necessary to further explore the time difference of factor flow on the convergence of urban-rural integration development in China. Here, the two-way fixed effect model of panel data were employed to investigate the situation in different regions in 2003–2011 and 2012–2020, respectively. The results are shown in Table 7.

As shown in Table 7, without considering the factor flow, the results of models (17) and (21) indicated that before and after the proposal of “promoting urban-rural integration” in 2012, the growth of urban-rural integration development demonstrated a convergence trend, and the subsequent convergence rate after 2012 is about 0.030 percentage points lower than that before 2012. Models (18)–(20), (22)–(24) considered the factor flow factors. We found significant differences in the impact of factor flow on the convergence of regional urban-rural integration and development around 2012. The convergence rate of urban-rural integration development before 2012 is generally higher than after 2012. At the same time, the interaction coefficient of capital flow, technology flow, and urban-rural integration development level also showed the opposite direction before and after 2012. However, the interaction coefficient of labor flow and urban-rural integration development was not significantly different before and after 2012.

### 6.2. Impulse Response Function Analysis

Impulse response function could directly reflect the dynamic interactive relationship and effect between variables and urban-rural integration development. To avoid orthogonalization dependence caused by the order of variables, VAR models of general impact response between variables and the development speed of urban-rural integration were established, respectively. The impact results of impulse response are shown in Figure 3.

Figure 3 demonstrated the impulse response function of urban-rural integration development caused by the impact of factor flow and its unit on urban-rural integration development since 2003. It was a short-term impact. As shown in Figure 3 (row 1, column 1), there was no increase in the development speed of urban-rural integration after the labor flow impacted urban-rural integration in the first year, while there was a slight increase soon. After that, the impact effect began to grow negatively in the second year and disappeared in the fifth year. As shown in Figure 3 (column 1 and column 2), when the development speed of urban-rural integration impacts itself in the first year, there is a growth in that year, and then the positive impact effect gradually weakens after fluctuations in the short term. As shown in Figure 3 (row 2, column 1), when the technology flow has an impact on the development of urban-rural integration, there is no negative growth in the year, and then there is a negative growth, and this impact effect weakens after reaching a shallow value in the second year. As shown in Figure 3 (row 2, column 2), the impact of capital flow on the development of urban-rural integration showed a “V” negative growth trend in the second year, and the impact effect disappeared in the fourth year.

### 6.3. Robustness Analysis

#### 6.3.1. Replace Interpreted Variable

To test the robustness of the above empirical results, the independent weight coefficient method is used to recalculate the regional urban-rural integration development index, which is substituted into the two-way fixed effect model of the panel data model for re-estimation. The results are shown in Table 8.

As shown in Table 8, when no other variables are added to the model (25), the regression coefficient of the initial urban-rural integration development was negative, indicating that there was absolute convergence of urban-rural integration development. After adding a series of regional control variables, the convergence rate increased by 0.084% (=0.116%–0.032%). After adding the interactive term of labor mobility and urban-rural integration development, the coefficient of urban-rural integration development in the base period and the coefficient of the interactive term were negative [34]. The convergence rate decreased by 0.014 percentage points. After adding the interaction term between technology flow and urban-rural integration development, the coefficient of urban-rural integration development in the base period and the coefficient of interaction term was negative, and the convergence rate decreased by 0.009 percentage points, indicating that factor flow might affect the growth and convergence of urban-rural integration development through interacting with urban-rural integration development.

#### 6.3.2. Rejection of Samples

Provinces and cities with the extreme growth trend of urban-rural integration development might have substantial heterogeneity and significantly impact the empirical results. Therefore, to overcome the possible impact of this situation, the top and bottom five provinces and cities in the urban-rural integration development were excluded, and the robustness of the above empirical conclusions was assessed. As shown in Table 9, when no other variables were added to the model (30), the regression coefficient of the initial urban-rural integration development was negative, indicating that there was absolute convergence of urban-rural integration development. After adding a series of regional control variables, the convergence rate increased by 0.006% (=0.123%–0.117%). After adding the interactive term of capital flow and urban-rural integration development, the coefficient of urban-rural integration development in the base period and the coefficient of the interactive term was positive, and the convergence rate increased by 0.048% (=0.171%–0.123%). After adding the interactive term of labor mobility and urban-rural integration development, the coefficient of urban-rural integration development level in the base period and the coefficient of the interactive term were negative. The convergence rate decreased by 0.003 percentage points. After adding the interactive term of technology flow and urban-rural integration development, the coefficient of urban-rural integration development level in the base period and the coefficient of the interactive term were negative. The convergence rate decreased by 0.003 percentage points. Factor flow affected the growing convergence of urban-rural integration development through the interaction effect with urban-rural integration development [35–37]. The capital flow positively affected the growing convergence of urban-rural integration development, while labor and technology flow showed a slowing effect on the growing convergence of urban-rural integration development. Higher labor and capital flows might slow down the convergence trend and widen the urban-rural integration development gap, further validating our conclusion's robustness.

## 7. Conclusions and Policy Recommendations

### 7.1. Conclusions

Based on the perspective of factor flow, we constructed the evaluation index system of urban-rural integration development using the panel data of 31 provinces in China from 2003 to 2020. The combined weighting model of GI and CRITIC were used to evaluate the regional urban-rural integration development. The impact of capital, labor, and technology factor flow on the convergence of urban-rural integration development was evaluated using the coefficient of variation and *β* convergence model. We further explored the time difference of factor flow on the growing convergence of regional urban-rural integration development and assessed the robustness. The main conclusions were as follows:

The growth of urban-rural integration development had an absolute convergence trend and tended to conditional convergence faster. The variation coefficient of urban-rural integration development and the regression coefficient of L. lny in model (1) was negative, indicating a definite convergence trend in urban-rural integration development. Furthermore, the estimated coefficient was still negative after controlling the time effect, indicating that the conclusion was stable. After introducing the variables such as fiscal decentralization (FD), rural financial services (Lnrfs), and per capita GDP (lnpgdp), the regression coefficients of L. lny were negative regardless of whether the time effect is controlled. The convergence rate of model (3) was 0.087 percentage points higher than that of model (1). Moreover, the rate of model (4) is 0.053 percentage points higher than that of model (2), implying that the growth of regional urban-rural integration development had the trend of absolute convergence, and it might tend to conditional convergence at a faster speed.

Nowadays, the capital flow has a positive effect on the convergence of urban-rural integration development, while labor flow and technology flow have a slowing effect on the convergence of urban-rural integration development. After adding the interaction term between capital flow and urban-rural integration development, the coefficient of urban-rural integration development in the base period was negative, whereas the coefficient of interaction term was positive, and the convergence rate increased. Capital flow positively affected the growth and convergence of urban-rural integration development. After adding the interactive term of labor mobility and urban-rural integration development, the coefficient of urban-rural integration development in the base period and the coefficient of the interactive term was negative, and the convergence rate decreased. After adding the interaction term between technology flow and urban-rural integration development, the coefficient of urban-rural integration development level in the base period and the coefficient of interaction term were negative, and the convergence speed also decreased. Labor and technology mobility slowed the growth and convergence of urban-rural integration development at this stage.

There were time differences in the impact of factor flow on the convergence of urban-rural integration development. The convergence rate of urban-rural integration development after 2012 was markedly slower than before. Before and after the proposal of “promoting urban-rural integration” in 2012, the growth of urban-rural integration development of provinces and cities in China showed a convergence trend, and the convergence rate was about 0.030 percentage points lower than before 2012. We also found significant differences in the impact of factor flow on the convergence of regional urban-rural integration and development around 2012. The convergence rate of urban-rural integration development before 2012 is higher than after 2012. Furthermore, the interaction coefficient of capital flow, technology flow, and urban-rural integration development also showed the opposite direction before and after 2012. However, the interaction coefficient of labor flow and urban-rural integration development had not changed before and after 2012.

### 7.2. Policy Suggestion

We should further promote the rural revitalization strategy and the two-way flow of urban and rural factors. The core of the rural revitalization strategy is talent revitalization. Establishing an institutional mechanism for the rational flow of urban and rural populations could attract rural and urban labor to stay in rural areas and start businesses to build rural areas. Establish and improve the introduction and training mechanism of professional farmers, cultivate new agricultural business entities, and improve the labor skills and quality of the rural population by establishing a talent training and exchange platform, strengthening the contact and cooperation between urban and rural talent markets, and establishing an information-sharing mechanism to provide institutional basis and policy guarantee for the rational flow and optimal allocation of urban and rural resources. Build the benefit-sharing mechanism for factor subjects, build a mechanism combining the complementary functions of the government and the market, and build the endogenous development mechanism of rural areas to promote the two-way flow of urban and rural factors, which guide the flow of production factors to rural areas.

Develop the financial allocation capacity of local governments and guide financial funds flow to rural areas. Financial support is the first element to develop a new countryside. Coordinating urban and rural development is a systematic project, which might not be realized only by market mechanism regulation. We should develop the positive guiding role of government funds, increase capital investment, leverage financial funds and social resources, and speed up the construction of a new countryside. We should increase fiscal expenditure on rural education, agricultural science, and technology; insist education as the foundation and technology as a means; improve the actual productivity of rural areas; and attract more talents to participate in rural construction. Establish and improve the government investment guarantee system to increase the public budget for agriculture and rural areas to fill the lack of agricultural and rural development. We should plan new financing ideas, strive for external progress, tap internal potential, and raise funds through multiple channels. Through the cross-regional transaction of land-saving indicators, more funds will be attracted to rural areas, and more rural people will share the urban development.

Focus on areas with slow urban-rural integration development and seek novel points. Promote the development of regional urban-rural integration, which tends to high-level convergence. We should promote the equalization of basic public services between urban and rural areas, improve the benefit-sharing mechanism for residents, and enable urban and rural residents to share the development of new urbanization. We might build basic public service facilities in urban and rural areas following unified allocation standards; further improve the security system for the elderly, the weak, the sick, and the disabled; and promote the integration of health care, old-age care, education, and employment. Promote the integration of urban and rural undertakings, increase investment in rural preschool education, and consolidate and enlarge teachers' teams. Insist overall consideration, individual breakthroughs, suit local conditions, fully consider the different stages of urban-rural integration development in different regions and the vast differences between diverse rural areas, and form a unique and practical development model of urban-rural integration.

## Figures and Tables

**Figure 1:** The nuclear density of urban-rural integration development in various regions. (source: made by authors).

**Figure 2:** Variation coefficient of urban-rural integrated development and factor flow. (source: made by authors).

**Figure 3:** Impulse response diagram. (source: made by authors).

**Table 1:** Evaluation index system of urban-rural integrated development.

Variable	Secondary index	Calculation method of secondary index	Index direction
Social integration	Urban and rural endowment insurance coverage	%	Positive
	Per capita health care expenditure ratio of urban and rural residents	—	Negative
	The ratio of urban and rural beds	—	Negative
	Employment ratio of urban and rural residents	—	Negative

Economic integration	Urban-rural consumption ratio	Rural residents = 1	Negative
	Urban-rural Engel coefficient ratio	Urban Engel coefficient/rural Engel coefficient	Positive
	Contribution of secondary and tertiary industries to GDP	%	Positive
	Difference between urban and rural fixed investment	Fixed asset investment (excluding farmers)/rural fixed-asset investment	Negative

Ecological integration	Forest coverage	Forest area/total land area/%	Positive
	Rural sanitary toilet penetration rate	%	Positive
	Urban and rural energy conservation and emission reduction	Total energy consumption/GDP 10000 tons of standard coal/100 million yuan	Negative
	Solid waste generation	10000 tons	Positive

Cultural integration	Township cultural station	Individual	Positive
	Comprehensive population coverage of rural radio programs	%	Positive
	The proportion of science and technology expenditure in financial expenditure	—	Positive
	Educational contrast coefficient	The difference in the proportion of urban and rural residents receiving primary and junior middle school education/10000	Negative

Spatial integration	Urban spatial expansion	The sown area of crops/built-up area/%	Positive
	Land urbanization level	Built-up area/total land area/%	Positive
	Highway mileage	Ten thousand kilometers	Positive
	Population urbanization level	Urban population/total population/%	Positive

**Table 2:** Descriptive statistics of variables.

Variables and description	Maximum	Minimum	Mean	SD	Median
Urban and rural endowment insurance coverage (%)	97.460	8.900	48.106	19.004	49.818
Per capita health care expenditure ratio of urban and rural residents	7.357	0.988	2.431	1.112	2.130
The ratio of urban and rural beds	49.062	0.029	3.383	8.777	0.870
Employment ratio of urban and rural residents	12.804	0.130	0.844	1.218	0.533
Urban-rural consumption ratio	7.200	1.474	2.784	0.759	2.665
Urban-rural Engel coefficient ratio	1.625	0.647	0.939	0.145	0.929
Contribution of secondary and tertiary industries to GDP (%)	99.807	65.784	88.845	6.030	89.172
Difference between urban and rural fixed investment	4085.607	5.156	117.418	403.283	34.300
Forest coverage (%)	68.411	0.430	32.299	18.137	34.310
Rural sanitary toilet penetration rate (%)	99.800	14.200	67.140	19.792	67.850
Urban and rural energy conservation and emission reduction	8.971	0.316	1.501	1.130	1.189
The output of solid waste (10000 tons)	61548.059	5.490	9183.874	9558.504	6312.410
Township cultural stations (PCs.)	4641.000	86.000	1099.593	773.800	1030.000
The comprehensive population coverage rate of rural radio programs (%)	100.000	77.781	95.939	4.385	97.250
The proportion of science and technology expenditure in financial expenditure	0.181	0.000	0.051	0.043	0.038
Educational contrast coefficient	0.674	0.007	0.182	0.115	0.153
Urban spatial expansion	1.413	0.006	0.425	0.265	0.418
Land urbanization level	15.070	0.006	1.684	2.660	0.729
Highway mileage (10000 km)	45.015	0.650	12.827	7.971	12.310
Population urbanization level	96.167	20.209	52.651	15.201	51.809
Labor mobility (LM)	2.821	0.061	1.015	0.720	0.823
Capital flows (CF)	2.468	0.419	1.003	0.301	0.931
Technology flow (TF)	3.312	0.060	1.016	0.735	0.887
Fiscal decentralization (FD)	23.117	0.000	1.211	3.178	0.324
Rural financial services (RFs yuan/person)	498139.573	150.615	23043.373	38193.529	16009.829
lnrfs	13.119	5.015	9.602	0.910	9.681
Per capita GDP (PGDP/yuan/person)	165002.285	3692.753	38434.218	27443.990	33461.355
lnpgdp	12.014	8.214	10.307	0.738	10.418

**Table 3:** Absolute convergence regression.

Variable	Model (1)	Model (2)	Model (3)	Model (4)
	Fixed effect	Fixed effect	Fixed effect	Fixed effect
L. lny	−0.036^*∗∗∗*^ (0.006)	−0.044^*∗∗∗*^ (0.014)	−0.123^*∗∗∗*^ (0.029)	−0.097^*∗∗∗*^ (0.017)
L. fd	—	—	−0.214^*∗∗∗*^ (0.049)	0.047 (0.052)
L. lnpgdp	—	—	0.018^*∗∗∗*^ (0.005)	0.023^*∗∗∗*^ (0.007)
L. lnrfs	—	—	0.005^*∗∗*^ (0.002)	0.003^*∗*^ (0.002)
Constant term	−0.004 (0.004)	−0.009 (0.012)	−0.278^*∗∗∗*^ (0.071)	−0.298^*∗∗∗*^ (0.070)
Province	*Y*	*Y*	*Y*	*Y*
Year	*N*	*Y*	*N*	*Y*
R^2^	0.046	0.454	0.120	0.481

Note. The values in brackets are the standard error of robustness. ^*∗∗∗*^, ^*∗∗*^, and ^*∗*^indicate significance at the level of 1%, 5%, and 10%, respectively.

**Table 4:** Conditional convergence regression results I (labor mobility).

Variable	Model (9)	Model (10)	Model (11)	Model (12)
	Fixed effect	Fixed effect	Fixed effect	Fixed effect
L. lny	−0.021 (0.013)	−0.087^*∗∗*^ (0.034)	−0.041^*∗∗*^ (0.017)	−0.091^*∗∗∗*^ (0.020)
L. lm	−0.027^*∗∗∗*^ (0.008)	−0.041^*∗∗∗*^ (0.011)	−0.027^*∗∗*^ (0.011)	−0.023^*∗∗*^ (0.011)
L. lny^*∗*^L. lm	−0.016^*∗*^ (0.009)	−0.032^*∗∗∗*^ (0.010)	−0.013^*∗*^ (0.008)	−0.012 (0.008)
L. fd	—	−0.257^*∗∗∗*^ (0.044)	—	0.012 (0.057)
L. lnpgdp	—	0.021^*∗∗∗*^ (0.005)	—	0.021^*∗∗∗*^ (0.007)
L. lnrfs	—	0.002 (0.001)	—	0.003^*∗∗*^ (0.002)
Constant term	0.023^*∗∗*^ (0.010)	−0.222^*∗∗∗*^ (0.073)	0.010 (0.014)	−0.258^*∗∗∗*^ (0.073)
Province	*Y*	*Y*	*Y*	*Y*
Year	*N*	*N*	*Y*	*Y*
R^2^	0.055	0.136	0.461	0.486

Note. The values in brackets are the standard error of robustness.^*∗∗∗*^, ^*∗∗*^, and ^*∗*^indicate significance at the level of 1%, 5%, and 10%, respectively.

**Table 5:** Conditional *β* convergence regression results II (capital flow).

Variable	Model (5)	Model (6)	Model (7)	Model (8)
	Fixed effect	Fixed effect	Fixed effect	Fixed effect
L. lny	−0.093^*∗∗∗*^ (0.025)	−0.218^*∗∗∗*^ (0.048)	−0.106^*∗∗∗*^ (0.028)	−0.149^*∗∗∗*^ (0.030)
L. cf	0.047^*∗∗∗*^ (0.016)	0.067^*∗∗∗*^ (0.022)	0.044^*∗∗∗*^ (0.016)	0.038^*∗∗*^ (0.016)
L. lny^*∗*^L. cf	0.058^*∗∗*^ (0.025)	0.085^*∗∗*^ (0.031)	0.049^*∗∗*^ (0.023)	0.045^*∗*^ (0.023)
L. fd	—	−0.241^*∗∗∗*^ (0.050)	—	0.013 (0.054)
L. lnpgdp	—	0.022^*∗∗∗*^ (0.006)	—	0.023^*∗∗∗*^ (0.007)
L. lnrfs	—	0.004^*∗*^(0.002)	—	0.002 (0.002)
Constant term	−0.050^*∗∗∗*^ (0.016)	−0.374^*∗∗∗*^ (0.085)	−0.063^*∗∗∗*^ (0.021)	−0.328^*∗∗∗*^ (0.071)
Province	Y	Y	Y	Y
Year	N	N	Y	Y
R^2^	0.059	0.142	0.465	0.488

*Note*. The values in brackets are the standard error of robustness. ^*∗∗∗*^, ^*∗∗*^, and ^*∗*^indicate significance at the level of 1%, 5%, and 10%, respectively.

**Table 6:** Conditional *β* convergence regression III (technology flow).

Variable	Model (13)	Model (14)	Model (15)	Model (16)
	Fixed effect	Fixed effect	Fixed effect	Fixed effect
L. lny	−0.026^*∗∗∗*^ (0.007)	−0.113^*∗∗∗*^ (0.030)	−0.037^*∗∗∗*^ (0.014)	−0.090^*∗∗∗*^ (0.017)
L. tf	−0.009 (0.006)	−0.013 (0.008)	−0.012^*∗∗*^ (0.006)	−0.013^*∗∗*^ (0.006)
L. lny^*∗*^L. tf	−0.021^*∗∗*^ (0.010)	−0.025^*∗*^ (0.013)	−0.022^*∗∗*^ (0.010)	−0.020^*∗∗*^ (0.010)
L. fd	—	−0.224^*∗∗∗*^ (0.049)	—	0.038 (0.053)
L. lnpgdp	—	0.020^*∗∗∗*^ (0.006)	—	0.026^*∗∗∗*^ (0.007)
L. lnrfs	—	0.004^*∗*^ (0.002)	—	0.002 (0.002)
Constant term	−0.001 (0.005)	−0.276^*∗∗∗*^ (0.077)	−0.006 (0.012)	−0.309^*∗∗∗*^ (0.071)
Province	*Y*	*Y*	*Y*	*Y*
Year	*N*	*N*	*Y*	*Y*
R^2^	0.055	0.129	0.460	0.486

*Note*. The values in brackets are the standard error of robustness. ^*∗∗∗*^, ^*∗∗*^and ^*∗*^indicate significance at the level of 1%, 5%, and 10%, respectively.

**Table 7:** The results of time differences.

Variable	2003–2011				2012–2020			
	Model (17)	Model (18)	Model (19)	Model (20)	Model (21)	Model (22)	Model (23)	Model (24)
L. lny	−0.080^*∗∗∗*^ (0.030)	−0.328^*∗∗∗*^ (0.063)	−0.140^*∗∗∗*^ (0.045)	−0.130^*∗∗∗*^ (0.038)	−0.060^*∗∗*^ (0.029)	0.044 (0.060)	−0.097^*∗∗*^ (0.041)	−0.092^*∗∗∗*^ (0.035)
L. cf	—	0.115^*∗∗∗*^ (0.040)	—	—	—	−0.052^*∗*^ (0.030)	—	—
L. lm	—	—	−0.021 (0.019)	—	—	—	−0.038 (0.024)	—
L. tf	—	—	—	−0.032^*∗*^ (0.017)	—	—	—	0.027^*∗∗*^ (0.012)
L. lny^*∗*^L. cf	—	0.159^*∗∗∗*^ (0.052)	—	—	—	−0.112^*∗∗*^ (0.045)	—	—
L. lny^*∗*^L. lm	—	—	−0.019 (0.019)	—	—	—	−0.005 (0.025)	—
L. lny^*∗*^L. tf	—	—	—	−0.050^*∗∗*^ (0.023)	—	—	—	0.055^*∗∗*^ (0.024)
L. fd	—	−0.126 (0.118)	−0.066 (0.128)	0.001 (0.113)	—	−0.027 (0.062)	0.014 (0.063)	0.024 (0.066)
L. lnpgdp	—	0.036^*∗∗*^ (0.014)	0.035^*∗∗*^ (0.015)	0.035^*∗∗*^ (0.014)	—	0.021 (0.013)	0.022^*∗*^ (0.013)	0.021 (0.013)
L. lnrfs	—	0.011^*∗∗*^ (0.005)	0.011^*∗∗*^ (0.005)	0.010^*∗*^ (0.005)	—	−0.003 (0.002)	−0.002 (0.003)	−0.002 (0.003)
Constant term	−0.039 (0.026)	−0.644^*∗∗∗*^ (0.136)	−0.505^*∗∗∗*^ (0.136)	−0.495^*∗∗∗*^ (0.132)	−0.015 (0.019)	−0.152 (0.136)	−0.220 (0.136)	−0.239^*∗*^ (0.137)
R^2^	0.246	0.335	0.312	0.324	0.644	0.670	0.655	0.656

*Note*. The values in brackets are the standard error of robustness. ^*∗∗∗*^, ^*∗∗*^, and ^*∗*^indicate significance at the level of 1%, 5%, and 10%, respectively.

**Table 8:** The results of robustness test I (replacement of explained variables).

Variable	Model (25)	Model (26)	Model (27)	Model (28)	Model (29)
L. lny	−0.032^*∗∗∗*^ (0.006)	−0.116^*∗∗∗*^ (0.029)	−0.200^*∗∗∗*^ (0.050)	−0.102^*∗∗∗*^ (0.031)	−0.107^*∗∗∗*^ (0.030)
L. cf	—	—	0.054^*∗∗∗*^ (0.019)	—	—
L. lm	—	—	—	−0.031^*∗∗*^ (0.012)	—
L. tf	—	—	—	—	−0.009 (0.007)
L. lny^*∗*^L. cf	—	—	0.072^*∗∗*^ (0.030)	—	—
L. lny^*∗*^L. lm	—	—	—	−0.026^*∗∗∗*^ (0.009)	—
L. lny^*∗*^L. tf	—	—	—	—	−0.020 (0.013)
L. fd	—	−0.174^*∗∗∗*^ (0.047)	−0.199^*∗∗∗*^ (0.046)	−0.206^*∗∗∗*^ (0.048)	−0.182^*∗∗∗*^ (0.047)
L. lnpgdp	—	0.016^*∗∗∗*^ (0.005)	0.020^*∗∗∗*^ (0.006)	0.019^*∗∗∗*^ (0.005)	0.017^*∗∗∗*^ (0.006)
L. lnrfs	—	0.005^*∗∗*^ (0.002)	0.004^*∗*^ (0.002)	0.005^*∗∗*^ (0.002)	0.005^*∗∗*^ (0.002)
Constant term	−0.001 (0.003)	−0.251^*∗∗∗*^ (0.068)	−0.334^*∗∗∗*^ (0.083)	−0.253^*∗∗∗*^ (0.068)	−0.250^*∗∗∗*^ (0.073)
R^2^	0.336	0.397	0.414	0.413	0.402

*Note*. The values in brackets are the standard error of robustness. ^*∗∗∗*^, ^*∗∗*^, and ^*∗*^indicate significant at the level of 1%, 5%, and 10%, respectively.

**Table 9:** The results of robustness test II (excluding some samples).

Variable	Model (30)	Model (31)	Model (32)	Model (33)	Model (34)
L.lny	−0.117^*∗∗∗*^ (0.026)	−0.123^*∗∗∗*^ (0.026)	−0.171^*∗∗∗*^ (0.037)	−0.120^*∗∗∗*^ (0.028)	−0.120^*∗∗∗*^ (0.025)
L. cf	—	—	0.039^*∗∗*^ (0.018)	—	—
L. lm	—	—	—	−0.039^*∗∗*^ (0.015)	—
L. tf	—	—	—	—	−0.026^*∗∗∗*^ (0.008)
L. lny^*∗*^L. cf	—	—	0.040 (0.026)	—	—
L. lny^*∗*^L. lm	—	—	—	−0.020^*∗*^ (0.010)	—
L. lny^*∗*^L. tf	—	—	—	—	−0.044^*∗∗∗*^ (0.013)
L. fd	—	0.077 (0.070)	0.051 (0.071)	0.003 (0.077)	0.036 (0.070)
L. lnpgdp	—	0.025^*∗∗∗*^ (0.009)	0.025^*∗∗∗*^ (0.009)	0.021^*∗∗*^ (0.009)	0.028^*∗∗∗*^ (0.009)
L. lnrfs	—	0.002 (0.002)	0.001 (0.002)	0.001 (0.002)	−0.001 (0.002)
Constant term	−0.071^*∗∗∗*^ (0.023)	−0.324^*∗∗∗*^ (0.080)	−0.363^*∗∗∗*^ (0.080)	−0.261^*∗∗∗*^ (0.083)	−0.336^*∗∗∗*^ (0.079)
R^2^	0.557	0.573	0.583	0.582	0.588

*Note*. The values in brackets are the standard error of robustness. ^*∗∗∗*^, ^*∗∗*^ and ^*∗*^,indicate significant at the level of 1%, 5%, and 10%, respectively.

## Data Availability

The data used to support the findings of this study are included in the article.
